# Comparative Analysis of the Anesthesia Effect of Cisatracurium Besylate and Mivacurium Chloride Otolaryngology Surgery

This article has been retracted.

**DOI:** 10.1155/2022/6192409

**Published:** 2022-07-18

**Authors:** Shibin Huang, Qi Li

**Affiliations:** ^1^Department of Otolaryngology, The Second Affiliated Hospital of Jiaxing University, No. 1518, Huancheng North Road, Jiaxing, Zhejiang 314000, China; ^2^Department of Anesthesiology, The Second Affiliated Hospital of Jiaxing Universit, No. 1518, Huancheng North Road, Jiaxing, Zhejiang 314000, China

## Abstract

**Objective:**

The aim is to investigate and compare the anesthesia effect of cisatracurium besylate and mivacurium chloride otolaryngology surgery.

**Materials and Methods:**

108 patients who underwent ENT surgery under general anesthesia in our hospital from November 2021 to March 2022 were recruited for retrospective analysis, in which patients in the experimental group A were anesthetized with cisatracurium besylate and patients in the experimental group B were anesthetized with mivacurium, and the anesthetic effects and recovery of the two groups were compared and analyzed.

**Results:**

There was no significant difference in mean arterial pressure, heart rate, and pulse oximetry levels between the two groups at the six time points of admission, anesthesia induction, intubation, end of operation, recovery of consciousness, and extubation (all *P* > 0.05). The train of four stimulation values at end of operation, recovery of consciousness, and extubation were significantly higher than those of the experimental group A (all *P* > 0.05). The recovery time of self-consciousness, extubation time, and eye-opening time of the experimental group B were significantly shorter than those of the experimental group A, and the occurrence of agitation was significantly less than that of the experimental group A (all *P* > 0.05). The total incidence of adverse conditions in the experimental group B was significantly lower than that in the experimental group A (*P* > 0.05).

**Conclusion:**

Compared with cisatracurium besylate in otolaryngology surgery, mivacurium chloride anesthesia offers a promising route with respect to less impact on hemodynamics, faster postoperative recovery, absence of the accumulation of neuromuscular blockade, less adverse reactions, and higher safety.

## 1. Introduction

Ear, nose, and throat surgery is one of the most common clinical procedures [1] and includes a variety of types, such as ear surgery, including otitis media surgery, hearing reconstruction surgery, and surgical treatment of vertigo; rhinologic surgery, including correction of nasal structures, turbinate hypertrophy surgery, sinusitis surgery, and nasal tumor surgery; and laryngeal surgery, including tonsil surgery, adenoid surgery, and hypopharyngeal tumor surgery. ENT surgery is characterized by relatively short duration and intense stimulation of the nerves and muscles of the patient's throat [2, 3]. Therefore, muscle relaxation and depth of anesthesia are highly demanded in otolaryngology surgery to ensure a quick anesthesia emergence after surgery. General anesthesia can be administered by tracheal intubation if the operation is difficult and if the intraoperative operation does not affect airway patency [4]; local anesthesia can be administered if the surgical site is superficial and the intraoperative operation does not affect airway patency. Local anesthesia is safer than general anesthesia or intravenous anesthesia [5].

There is convincing observational evidence supporting that among the anesthetic drugs, cisatracurium besylate has a significant muscle relaxant effect, and mivacurium chloride has fewer side effects. Cisatracurium besylate for injection, a white loose lump or powder with molecular formula of C_65_H_82_N_2_O_18_S_2_, is a moderate-acting, nondepolarizing skeletal muscle relaxant with an isoquinolinium benzyl ester structure and a neuromuscular blocker [6, 7]. Human clinical studies have shown that cisatracurium besylate binds to cholinergic receptors on the motor endplate to antagonize the action of acetylcholine, resulting in a competitive neuromuscular blockade [8, 9]. At present, it is predominantly used for surgery and other operations in intensive care treatment. Due to the characteristics of relaxing skeletal muscles and convenience to perform tracheal intubation and mechanical ventilation, it is thus used clinically as an adjuvant drug for general anesthesia or as a sedative in intensive care [10, 11]. Mivacurium chloride [12], a gray-white solid with a molecular formula of C_58_H_80_C_l2_N_2_O_14_, is a short-acting benzylisoquinoline nondepolarizing muscle relaxant [13]. Clinically, it is majorly used in short-term surgical procedures and can be used as an adjuvant drug for general anesthesia during tracheal intubation and mechanical ventilation [14]. For example, mivacurium chloride is commonly used as the first-choice anesthetic in cystoscopic resection of bladder cancer [15]. Available findings indicate that it is the most effective and selective nondepolarizing inotropic drug available clinically, with the advantages of rapid onset of action, rapid recovery, few side effects, no drug accumulation, no adverse effects on the autonomic nervous system and cardiovascular system, and elimination half-life [16, 17]. However, there are few studies of clinical application of mivacurium chloride minor surgery, such as otolaryngology surgery, and there are also few related studies comparing the anesthetic effects of cisatracurium besylate and mivacurium chloride. To address the gap, this study was to investigate and compare the anesthesia effects of cisatracurium besylate and mivacurium chloride otolaryngology surgery, aiming to provide new ideas and routes for anesthesia.

## 2. Materials and Methods

### 2.1. General Information

A total of 108 patients who underwent otolaryngology surgery under general anesthesia in our hospital from November 2021 to March 2022 were retrospectively analyzed and were evenly allocated into an experimental group A and an experimental group B. This study has been reviewed and approved by the Medical Ethics Committee of the Second Affiliated Hospital of Jiaxing University, approval no. 9799/31.

### 2.2. Inclusion and Exclusion Criteria

#### 2.2.1. Inclusion Criteria

Inclusion criteria are as follows: all were graded I-II by the American Society of Anesthesiologists (ASA); the preoperative acid-base balance and water and electrolyte stability; and the patients and their families were aware of the study and signed written consent form voluntarily.

#### 2.2.2. Exclusion Criteria

Exclusion criteria are as follows: patients combined with abnormal heart, liver, and kidney functions; patients combined with blood diseases or coagulation disorders; and research related drug allergies.

## 3. Methods

Both groups of patients underwent routine anesthesia induction after entering the operating room. 1-2 *μ*g/kg remifentanil (approval no. H20030200, Yichang Renfu Pharmaceutical Co., Ltd.), 1-2 mg/kg propofol (approval no. H20051843, Sichuan Guorui Pharmaceutical Co., Ltd.), and 0.05–0.10 mg/kg midazolam (approval no. H20113433, Jiangsu Enhua Pharmaceutical Co., Ltd.) were intravenously administered 30 min before operation. After the patient lost consciousness, the closed-loop muscle relaxant injection system was opened, and muscle relaxant drugs were given.

The patients in the experimental group A were anesthetized via cisatracurium besylate (approval no. H20060927, Dongying Pharmaceutical Co., Ltd.) with an induction dose of 0.15 mg/kg and a maintenance rate of 0.1 mg/(kg·h); patients in the experimental group B were given mivacurium chloride (approval no. H20100454, GlaxoSmithKline Manufacturing S.P.A) for anesthesia with an induction dose of 0.2 mg/kg and a maintenance rate of 0.15% mg/(kg h). Both groups were intubated through the orotracheal tube when the maximum inhibition was reached, and then, the anesthesia machine was connected and relevant parameters were adjusted. The respiratory rate was 12 times/min, the tidal volume was 8 ml/kg, and the inspiratory ratio was 1 : 2.

During the maintenance period, propofol + remifentanil + sevoflurane was given as follows: propofol 2 mg/kg was slowly pushed, and the bronchoscope was introduced when breathing and circulation were stable. During the operation, propofol was added intermittently depending on the patient's response, and anesthesia was maintained by inhalation of sevoflurane; the dosage of remifentanil was adjusted according to the hemodynamics and respiratory rate, with an increase or decrease of 0.025 *μ*g/(kg·min) each time. Inhalation was stopped 20 minutes before the end of the operation, and no muscle relaxant antagonist was used after the operation.

### 3.1. Observation Indicators

① Monitoring devices are used to continuously monitor and record mean arterial pressure (MAP), heart rate (HR), and pulse oximetry (SpO_2_). The patients' hemodynamic parameters are monitored at admission, during induction of anesthesia, during intubation, at the end of the procedure, at recovery of consciousness, and at extubation.

② Train of four (TOF) stimulations: the TOF values of the above six time points in the two groups of patients were compared.

③ Recovery situation: the recovery time of self-consciousness, extubation time, and eye-opening time and the occurrence of agitation in the two groups from the beginning of surgical anesthesia to 1 hour after extubation were compared between the two groups.

④ Adverse reactions: the occurrence of adverse reactions in the two groups after operation, including residual muscle relaxation, hypotension, bronchospasm, skin flushing, nausea, and vomiting, were observed and compared.

### 3.2. Statistical Analysis

The SPSS 22.0 software was used to process the data. The enumeration data (*n* (%)) and measurement data (*x* ± *s*) were examined via the chi-square and *t* tests, respectively. *P* < 0.05 was considered statistically significant.

## 4. Results

### 4.1. General Information

In the experimental group A, there were 28 males and 26 females, aged 25–61 years, with an average of 40.28 ± 4.87 years, and a BMI of 22–25 kg/m^2^, with an average of 23.84 ± 1.21 kg/m^2^. In the experimental group B, there were 27 females, aged 23–64 years, with an average age of 40.88 ± 3.97 years, and a BMI of 22–26 kg/m^2^, with an average of 23.98 ± 1.08 kg/m^2^. The baseline data were comparable between the two groups of patients (Table 1).

### 4.2. Hemodynamics

There was no significant difference in MAP, HR, and SpO_2_ levels between the two groups at the six time points of admission, anesthesia induction, intubation, end of operation, recovery of consciousness, and extubation (all *P* < 0.05) (Tables 2–4).

### 4.3. TOF Value

The TOF values were similar at the three time points of admission, anesthesia induction, and intubation between the two groups of patients (all *P* > 0.05); whereas, TOF values (36.81 ± 8.23, 79.87 ± 2.56, and 90.62 ± 6.29) at end of operation, recovery of consciousness, and extubation were significantly higher than those of the experimental group A (25.18 ± 4.07, 59.89 ± 5.02, and 80.86 ± 3.68) (all *P* < 0.05) (Table 5).

### 4.4. Recovery

The recovery time of self-consciousness, extubation time, and eye-opening time (4.87 ± 1.02, 7.68 ± 1.41, and 9.82 ± 1.65) of the experimental group B were significantly shorter than those of the experimental group A (12.18 ± 1.34, 20.85 ± 6.32, and 25.94 ± 5.65), and the occurrence of agitation (3.70%) was significantly less than that of the experimental group A (20.37%) (all *P* < 0.05) (Table 6).

### 4.5. Adverse Reactions

In the experimental group A, there were 2 cases (3.70%) of residual muscle relaxation, 1 case of hypotension (1.85%), 2 cases of skin flushing (3.70%), 4 cases of nausea and vomiting (7.41%), and 0 case of residual muscle relaxation (0.00%); in the experimental group B, 0 case of hypotension (0.00%), 0 cases of skin flushing (0.00%), and 1 case of nausea and vomiting (1.85%), and the total incidence of adverse conditions in the experimental group B (1.85%) was significantly lower than that in the experimental group A (16.67%) (*P* < 0.05) (Table 7).

## 5. Discussion

Anesthesia for ENT surgery is one of the keys to ensure successful surgery. Surgical anesthesia requires the selection of appropriate anesthetic methods and drugs [18–20]. As tracheal intubation and surgery are accompanied by varying degrees of anesthesia and muscle relaxation, the inevitable residual neuromuscular blockade after surgery possesses a challenge to surgical anesthesia. The choice of drug or method should take into account the patient's psychological and physiological status to ensure good anesthetic outcomes while controlling the magnitude of hemodynamic fluctuations [21].

Among the current clinical anesthetics, both cisatracurium besylate and mivacurium chloride are good choices, and each has its own advantages. For example, the former has a remarkable muscle relaxation effect [22], while the latter is associated with fewer side reactions [23]. Currently, it remains controversial which is more effective. In line with our hypotheses, we found that there was no significant difference in MAP, HR, and SpO_2_ levels between the two groups at the six time points of admission, anesthesia induction, intubation, end of operation, recovery of consciousness, and extubation; and TOF values were similar at the three time points of admission, anesthesia induction, and intubation between the two groups of patients; whereas, TOF values at end of operation, recovery of consciousness, and extubation were significantly higher than those of the experimental group A. However, this interpretation is supported by the fact that the rapid onset of action of mivacurium chloride and the absence of significant neuromuscular blockade accumulation as demonstrated by monitoring with a muscle relaxation monitor facilitated a reduction in depth of anesthesia towards the end of the procedure [23]. Possible explanations are that this study required a closed-loop myorelaxant injection, which allows for effective individualization of dosing and helps to avoid drug wastage due to long-term myorelaxant use; mivacurium chloride is a synthetic diquaternary compound with two ester bonds and therefore has a rapid onset of action and a short duration of action with an elimination half-life of 2-3 minutes, consistent with previous studies [24].

Also, in keeping with our hypotheses, we found that the recovery time of self-consciousness, extubation time, and eye-opening time of the experimental group B were significantly shorter than those of the experimental group A, and the occurrence of agitation was significantly less than that of the experimental group A. This would suggest that the recovery of muscle contraction function in patients receiving mivacurium chloride after otolaryngology surgery was better than using cisatracurium besylate. It is assumed that cisatracurium besylate is a nondepolarizing muscle relaxant due to its similar metabolism and myorelaxant effect to atracurium, although it has fewer side effects on the human cardiovascular system but a higher muscle relaxant effect [25, 26]; mivacurium chloride is a diquaternary ammonium compound that can be synthesized as a substitute for succinylcholine. It is a short-acting benzylisoquinoline nondepolarizing muscarinic agent with short duration of action, rapid onset of action, rapid metabolism, no accumulation, and rapid recovery [27, 28]. It has relatively few autonomic and cardiovascular side effects. After discontinuation of the drug, the patient can regain muscle tone naturally within a short period of time [29].

As previously noted, both cisatracurium besylate and micuronium anesthesia will cause different degrees of damage to patients and lead to adverse reactions. The adverse effect profile of micuronium anesthesia is related to histamine release and dose, but can be reduced by splitting or adjusting the time of administration. It is also of interest that the treatment in the experimental group B was associated with lower incidence of adverse reactions. We suggest this is perhaps because the application of mivacurium chloride anesthesia can reduce the occurrence of residual muscle relaxation during the recovery period and after recovery, playing a positive role on both mental and physical recovery of patients after surgery, and the data support findings of the trail of Farhan et al. [30].

Adverse reactions that have been recorded with atracurium cisbenzoate include skin flushing or rash, bradycardia, hypotension, and bronchospasm. Allergic reactions of varying degrees of severity can be observed following the use of neuromuscular blocking agents [31]. In rare cases, severe allergic reactions have been reported when this product is combined with one or more anesthetic agents [32]. Myasthenia and/or myopathy have been reported in severely ill patients in intensive care units after prolonged use of muscle relaxants [33]. Most patients received concomitant steroid preparations, and these have occasionally been reported following the use of this product, but the causal relationship has not been established [34].

## 6. Conclusion

To sum up, compared with cisatracurium besylate in otolaryngology surgery, mivacurium chloride anesthesia offers a promising route with respect to less impact on hemodynamics, faster postoperative recovery, absence of the accumulation of neuromuscular blockade, less adverse reactions, and higher safety. Overall, it merits widespread clinical application. However, there are many limiting factors in the experiment. First, comparisons between multiple time points in our experiments required a one-way ANOVA. Second, many indicators are related to the follow-up time, and we need to conduct more in-depth analysis after follow-up investigations in follow-up studies.

## Figures and Tables

**Table 1:** Baseline data ($\bar{x}\pm s$).

Groups	*n*	Male	Female	Age (years)	Mean age (years)	BMI	Mean BMI
Experimental group A	54	28	26	25–61	40.28 ± 4.87	22–25	23.84 ± 1.21
Experimental group B	54	27	27	23–64	40.88 ± 3.97	22–26	23.98 ± 1.08
*T*	—	—	—	—	0.341	—	0.521
*P*	—	—	—	—	0.798	—	0.545

**Table 2:** Comparison of hemodynamics between the two groups of patients ($\bar{x}\pm s$).

Groups	*n*	Upon admission			Anesthesia induction		
		MAP (mmHg)	HR (times/min)	SpO_2_ (%)	MAP (mmHg)	HR (times/min)	SpO_2_ (%)
Experimental group A	54	103.12 ± 9.38	82.38 ± 7.21	97.73 ± 11.11	100.98 ± 7.21	79.82 ± 8.41	98.21 ± 10.29
Experimental group B	54	102.61 ± 10.33	83.54 ± 9.12	96.74 ± 11.98	101.01 ± 12.04	80.18 ± 10.63	98.11 ± 10.82
*t*	—	0.496	0.274	0.297	0.473	0.288	0.354
*P*	—	0.684	0.688	0.754	0.692	0.726	0.594

**Table 3:** Comparison of hemodynamics between the two groups of patients ($\bar{x}\pm s$).

Groups	*n*	Intubation			End of operation		
		MAP (mmHg)	HR (times/min)	SpO_2_ (%)	MAP (mmHg)	HR (times/min)	SpO_2_ (%)
Experimental group A	54	115.41 ± 6.02	74.53 ± 6.21	99.65 ± 14.52	109.65 ± 9.11	70.41 ± 8.01	99.51 ± 10.02
Experimental group B	54	112.88 ± 9.63	75.42 ± 11.02	99.81 ± 10.32	105.12 ± 7.63	70.52 ± 9.45	99.98 ± 11.41
*t*	—	0.357	0.294	0.456	0.461	0.213	0.323
*P*	—	0.702	0.813	0.582	0.598	0.814	0.757

**Table 4:** Comparison of hemodynamics between the two groups of patients ($\bar{x}\pm s$).

Groups	*n*	Recovery of consciousness			Extubation		
		MAP (mmHg)	HR (times/min)	SpO_2_ (%)	MAP (mmHg)	HR (times/min)	SpO_2_ (%)
Experimental group A	54	113.52 ± 8.09	82.63 ± 5.19	94.08 ± 17.62	117.62 ± 7.68	87.49 ± 3.92	95.01 ± 13.52
Experimental group B	54	114.17 ± 8.87	83.65 ± 7.62	98.46 ± 9.44	118.21 ± 10.39	86.69 ± 8.11	96.34 ± 9.61
*t*	—	0.024	0.276	0.268	0.703	0.058	0.123
*P*	—	0.997	0.683	0.759	0.484	0.996	0.624

**Table 5:** Comparison of TOF values between the two groups of patients ($\bar{x}\pm s$).

Groups	*n*	Upon admission	Anesthesia induction	Intubation	End of operation	Recovery of consciousness	Extubation
Experimental group A	54	99.36 ± 12.68	99.15 ± 10.68	0.00 ± 0.00	25.18 ± 4.07	59.89 ± 5.02	80.86 ± 3.68
Experimental group B	54	99.54 ± 12.05	99.24 ± 6.88	0.00 ± 0.00	36.81 ± 8.23	79.87 ± 2.56	90.62 ± 6.29
*t*	—	0.075	0.068	0.000	18.451	14.412	19.002
*P*	—	0.932	0.944	1.000	＜0.001	＜0.001	＜0.001

**Table 6:** Comparison of the recovery of the two groups of patients ($\bar{x}\pm s$, %).

Groups	*n*	Self-consciousness recovery time (min)	Extubation time (min)	Eye-opening time (min)	Cases of agitation occurs (*n*)
Experimental group A	54	12.18 ± 1.34	20.85 ± 6.32	25.94 ± 5.65	11 (20.37)
Experimental group B	54	4.87 ± 1.02	7.68 ± 1.41	9.82 ± 1.65	2 (3.70)
*t*	—	13.254	15.667	19.024	8.945
*P*	—	＜0.001	＜0.001	＜0.001	0.002

**Table 7:** Comparison of adverse reactions in the two groups of patients (%).

Groups	*n*	Muscle relaxation remnants	Low blood pressure	Flushing of the skin	Nausea and vomiting	Total incidence
Experimental group A	54	2 (3.70)	1 (1.85)	2 (3.70)	4 (7.41)	9 (16.67)
Experimental group B	54	0 (0.00)	0 (0.00)	0 (0.00)	1 (1.85)	1 (1.85)
*t*	—	8.804				
*P*	—	0.003				

## Data Availability

The data generated or analyzed during this study are included within the article.
